# Model of Epidemic Kinetics with a Source on the Example of Moscow

**DOI:** 10.1155/2022/6145242

**Published:** 2022-02-18

**Authors:** Andrey V. Borovsky, Andrey L. Galkin

**Affiliations:** ^1^Department of Mathematical Methods and Digital Technologies, Baikal State University, 664003 Irkutsk, Russia; ^2^Department of High-Power Lasers, Prokhorov General Physics Institute of the Russian Academy of Sciences, 119991 Moscow, Russia

## Abstract

A new theoretical model of epidemic kinetics is considered, which uses elements of the physical model of the kinetics of the atomic level populations of an active laser medium as follows: a description of states and their populations, transition rates between states, an integral operator, and a source of influence. It is shown that to describe a long-term epidemic, it is necessary to use the concept of the source of infection. With a model constant source of infection, the epidemic, in terms of the number of actively infected people, goes to a stationary regime, which does not depend on the population size and the characteristics of quarantine measures. Statistics for Moscow daily increase in infected is used to determine the real source of infection. An interpretation of the waves generated by the source is given. It is shown that more accurate statistics of excess mortality can only be used to clarify the frequency rate of mortality of the epidemic, but not to determine the source of infection.

## 1. Introduction

The situation with the epidemic of the coronavirus infection dictates the use of laser physics methods to describe the development of the epidemic. Elements of a physical model of the kinetics of atomic level populations [1] for active media of laser systems can be used to construct an epidemic model. The four elements are as follows: states and their populations, rates of transitions between states, a time integral operator, and a source of influence. As applied to the description of the epidemic, the population of the settlement (a set of atoms) is divided into groups (atoms are in different states) as follows: healthy nonimmune, infected, recovered, and fatal members of the population. Between these states, similarly to laser physics, transitions take place at their own speeds. The concepts of rates of infection, recovery, and transition to the lethal group are introduced. The rates of emptying of the states of the atom are equal to the reciprocal of the decay time of the states; therefore, following a physical analogy, in epidemic kinetics, the rate of recovery is equal to the reciprocal of the time period of the disease, the same with the fatal outcome. The integral operator in the kinetics of populations realizes the spatial connection of atoms; in the model of epidemic kinetics, the integral operator in time takes into account the infection of members of the population during the incubation period of the disease and mortality outside the incubation period. The time integral operator of epidemic kinetics is reduced to lagging terms, which distinguishes it from the classical SIR model (literally means susceptible-infected-recovered).

Epidemic modeling work is divided into two types. The first [3–7] uses a balanced approach applicable for locality or region. In [4], a 7-fraction model of the hepatitis B epidemic is considered. In [5, 6], 6-fraction (SEIARD and SEIAHR) COVID-19 models were studied. In [7], a model with vaccination of the population (SVEAIR) is presented.

The second approach [8] further describes the spatial propagation epidemic. Thus, the mathematical model of the Baroyan-Rvachev influenza epidemic [9, 10] is classified as epidemic dynamics, since it can describe the undulating spread of the epidemic between cities when taking into account the passenger traffic (the model is similar to the equations of hydrodynamics). Moreover, all models do not take into account the source of infection [11]. The need to take into account the source of infection is indicated in [2]. Only in this case is it possible to build adequate epidemic models that coincide with real statistics.

The aim of this work is to investigate the role of a nonstationary source of infection in delayed epidemic kinetics. In this case, a mathematical model of the epidemic is applied, using elements of physical models of laser physics associated with the description of active laser media.

## 2. Numerical Investigations of the Equations of Epidemic Kinetics with Delay with a Constant Source

The model is constructed on the basis of balanced equations, similar to the physical problem of atomic level kinetics.

Let us first consider the model of epidemic kinetics without taking into account the process of vaccination of citizens. For example, in Russia, it was possible not to take into account the vaccination of the population until May 2021. The model considers the development over time of an epidemic of viral infection in a locality whose population is a constant value *N*_0_. The population of the locality is divided into 4 categories: *N*_1_, healthy members of the population who do not have immunity; *N*_2_, infected; *N*_3_, acquired immunity (recovered); and *N*_4_, members of the population who fell into the lethal group (died) during the entire epidemic.

For a closed population, the law of population conservation is fulfilled

(1) $$\begin{array}{c} \overset{4}{\underset{i=1}{\sum }}N_{i}=N_{0}. \end{array}$$

To fulfill (1), it is necessary that the natural birth rate is equal to the natural mortality of the population, and the speed of departure of the population is equal to the speed of arrival in the locality. For example, the population of the city of Irkutsk has remained at a constant level for 30 years. In addition, the time of epidemic development *T*~2-3 years is significantly less than the time of migration processes for settlements such as an average city. All the above values depend on time *N*_*i*_(*t*), and *N*_0_ is a constant value.

The characteristics of the epidemic development are “global statistics variables,” which are called the number of infected members of the population since the beginning of the epidemic *N*_−_(*t*), the number of recovered members of the population since the beginning of the epidemic *N*_+_(*t*), and the number of the lethal group since the beginning of the epidemic *N*_*c*_(*t*). It is easy to see that the values *N*_+_(*t*) and *N*_*c*_(*t*) coincide with *N*_3_(*t*) and *N*_4_(*t*) in the epidemic kinetic model, which does not take into account vaccination.

(2) $$\begin{array}{c} N_{+}\left(t\right)\equiv N_{3}\left(t\right),N_{c}\left(t\right)\equiv N_{4}\left(t\right). \end{array}$$

The variable of global infection statistics is related to the parameters of epidemic kinetics as follows:

(3) $$\begin{array}{c} N_{1}\left(t\right)+N_{-}\left(t\right)=N_{0}. \end{array}$$

From here, we get

(4) $$\begin{array}{c} N_{-}\left(t\right)=N_{2}\left(t\right)+N_{3}\left(t\right)+N_{4}\left(t\right). \end{array}$$

We see that the number of infected persons can be expressed in terms of global statistic variables

(5) $$\begin{array}{c} N_{2}\left(t\right)=N_{-}\left(t\right)-N_{+}\left(t\right)-N_{c}\left(t\right). \end{array}$$

Let us write down an expression for the rate of change in the number of infected persons

(6) $$\begin{array}{c} \frac{dN_{2}\left(\text{t}\right)}{dt}=\frac{dN_{-}\left(t\right)}{dt}-\frac{dN_{+}\left(t\right)}{dt}-\frac{dN_{c}\left(t\right)}{dt}=\frac{dN_{-}\left(t\right)}{dt}-\frac{dN_{3}\left(t\right)}{dt}-\frac{dN_{4}\left(t\right)}{dt}. \end{array}$$

The first term in the right part describes the rate of infection of members of the population; the second, the rate of recovery; and the third, the rate of transition to the lethal group. The rate of infection will be determined by the number of members of the population who are in the latent incubation period of infection *τ* and those who carry the infection in an asymptomatic manner, i.e., undetected carriers of infection

(7) $$\begin{array}{c} \frac{dN_{-}\left(t\right)}{dt}=k^{-}\left(\int_{t-\tau }^{t}\frac{dN_{-}\left(t^{\prime }\right)}{dt^{\prime }}K\left(t-t^{\prime }\right)dt^{\prime }+\gamma_{1}\int_{0}^{t-\tau }\frac{dN_{-}\left(t^{\prime }\right)}{dt^{\prime }}K\left(t-t^{\prime }\right)dt^{\prime }\right). \end{array}$$

*K*(*t* − *t*′)− is the core of the integral operator, which describes the decrease in infected individuals over time. The type of model function *K*(*t*) can be selected as

(8) $$\begin{array}{c} K\left(t\right)=\exp\left[-{\left(\frac{t}{\tau_{+}}\right)}^{2}\right]. \end{array}$$

The real form of the kernel of the integral operator *K*(*t*) should be determined by comparison with the statistics of the epidemic.

Assuming *K*(*t*) = 1, which somewhat overestimates the number of persons transmitting the infection, integrals in (7) are revealed and lagging terms appear

(9) $$\begin{array}{c} \frac{dN_{-}\left(t\right)}{dt}=k^{-}\left(N_{-}\left(t\right)-\left(1-\gamma_{1}\right)N_{-}\left(t-\tau \right)\right). \end{array}$$

The rate of recovery of infected citizens is proportional to the number of infected at a given time

(10) $$\begin{array}{c} \frac{dN_{3}\left(t\right)}{dt}=k^{+}N_{2}\left(t\right). \end{array}$$

The rate of death is determined by the number of infected persons, taking into account the delay in the development of the disease

(11) $$\begin{array}{c} \;\frac{dN_{4}\left(t\right)}{dt}=k^{c}N_{2}\left(t-\tau \right). \end{array}$$

Given the large volume of testing of the population and the isolation of asymptomatically ill persons in the city of Moscow, it is possible to put *γ*_1_≅0. A significant change in the values *N*_3_(*t*) and *N*_4_(*t*) occurs at times *t* > 3*τ*, while *N*_2_(*t*) is sensitive to changes at times *t* < *τ*. Therefore,

(12) $$\begin{array}{c} N_{-}\left(t\right)-\left(1-\gamma_{1}\right)N_{-}\left(t-\tau \right)≅N_{-}\left(t\right)-N_{-}\left(t-\tau \right)≅N_{2}\left(t\right)-N_{2}\left(t-\tau \right). \end{array}$$

As a result, we come to the following modification of the epidemic kinetics model

(13) $$\begin{array}{c} \frac{dN_{1}\left(t\right)}{dt}=-k^{-}\left|N_{2}\left(t\right)-N_{2}\left(t-\tau \right)\right|-А,\frac{dN_{2}\left(\text{t}\right)}{dt}=k^{-}\left|N_{2}\left(t\right)-N_{2}\left(t-\tau \right)\right|-k^{+}N_{2}\left(t\right)-k^{c}N_{2}\left(t-\tau \right)+А,\frac{dN_{3}\left(t\right)}{dt}=k^{+}N_{2}\left(t\right),\frac{dN_{4}\left(t\right)}{dt}=k^{c}N_{2}\left(t-\tau \right). \end{array}$$

The equations with lagging terms in (13) are not first-order differential equations. The delayed term *N*_2_(*t* − *τ*) can be decomposed into a Taylor series. At the same time, higher-order derivatives appear. For example, in [2], the second equation in system (13) was reduced to an ordinary differential equation of the second order, which had a bell-shaped solution of the epidemic wave type.

Here, the coefficients *k*^−^, *k*^+^, and *k*^*c*^ have the dimension of frequency, i.e., the inverse time, which is measured in days. All data in epidemic statistics are presented per day. The number of different categories of the population is determined in persons.

The value *A* represents the rate of quasistationary permanent sources of infection. The value of *A* can change slowly. However, the time of such change is significantly longer than the inverse frequencies present in the model and the time of the latent incubation period of infection development

(14) $$\begin{array}{c} T\gg {\left(k^{-}\right)}^{-1},{\left(k^{+}\right)}^{-1},{\left(k^{c}\right)}^{-1},\tau . \end{array}$$

We note the following circumstance, which negates the choice of a nonstationary model for epidemic kinetics. Numerical calculations have shown that the unsteady mode of epidemic development occurs only at the initial stage within 90-100 days. All the subsequent time, the epidemic develops in a quasistationary mode, which weakly depends on the expression for the rate of infection. (Such modes are well known in laser physics. They arise for long or generally stationary pulses of pumping the active medium of the laser *A*(*t*) ≈ Const.)

For the COVID-19 disease caused by the SARS-CoV-2 coronavirus (as opposed to, for example, the flu), we take the recovery time of the *τ*^+^ = 15 Day, then the recovery rate is the reciprocal *κ*^+^ = 1/15Day^−1^. The frequency of death is similar to *κ*^*c*^ = 1/50Day^−1^. The duration of the incubation period of the *τ* = 7 Day and the frequency of infection are represented by the expression

(15) $$\begin{array}{c} \kappa^{-}\left(t\right)=p\left(t\right)\dot{\Delta n}\left(t\right)=p\left(t\right){\dot{\Delta n}}_{0}\left(t\right)\frac{N_{1}\left(t\right)}{N_{0}},\overset{4}{\underset{i=1}{\sum }}N_{i}\left(t\right)=N_{0}. \end{array}$$

Expression (15) takes into account that the rate of contact of an infected person with uninfected persons should decrease as the epidemic proceeds in proportion to the share of healthy noninfected persons in the population of the locality

(16) $$\begin{array}{c} \dot{\Delta n}\left(t\right)={\dot{\Delta n}}_{0}\left(t\right)\frac{N_{1}\left(t\right)}{N_{0}}. \end{array}$$

Here, ${\dot{\Delta n}}_{0}\left(t\right)-$ is the rate of contacts with all persons who were not ill and recovered.

The following expressions are used for the frequency of contacts and the likelihood of infection:

(17) Δn˙t=Δn˙in;0<t<t′Δn˙in−Δn˙in−Δn˙ft−t′t′′−t′;t′≤t≤t′′,Δn˙f;t′′≤tpt=pin;0<t<t′,pin−pin−pft−t′t′′−t′pf;t′′≤t.;t′≤t≤t′′,

Formula (17) describes the smooth introduction of sanitary standards. Designations ${\dot{\Delta n}}_{\text{in}},{\dot{\Delta n}}_{f}$ and *p*_in_, *p*_*f*_ correspond to the initial and final values of the rate of contacts and the possibility of infection. The calculations used the values$\;{\dot{\Delta n}}_{\text{in}}=30,{\dot{\Delta n}}_{f}=20$ and *p*_in_ = 0.01, *p*_*f*_ = 0.005.

The statement of problem (13) should be supplemented by the condition of nonnegativity of the sought functions and by the initial conditions, for example,

(18) $$\begin{array}{c} N_{i}\left(t\right)\geq 0,i=1,..4,\;N_{1}\left(0\right)=N_{0},\;N_{2}\left(0\right)=1,\;N_{3}\left(0\right)=0,\;N_{4}\left(0\right)=0. \end{array}$$

To numerically solve the problem of epidemic kinetics (8)–(12), a difference scheme is used, a feature of which is memorizing the prehistory to a given moment *t* (for example, with a step of 0.1 days) of already obtained functions *N*_*i*_(*s*), *s* ≤ *t*.

In the approximation  *N*_1_(*t*) ≈ *N*_0_, the *κ*^−^(*t*) in (15) does not depend on  *N*_1_(*t*) and the second equation in (13) becomes independent, and the remaining components are determined through this solution  *N*_2_(*t*).

In the approximation *N*_1_(*t*) ≈ *N*_0_ at small times without taking into account the delay from the second equation of system (13),

(19) $$\begin{array}{c} \frac{dN_{2}}{dt}\left(t\right)=\left(\kappa^{-}\left(0\right)-\kappa^{+}\right)N_{2}\left(t\right)+А. \end{array}$$

We get the analytical expression

(20) $$\begin{array}{c} N_{2}\left(t\right)=N_{2}\left(0\right)e^{\left(k^{-}\left(0\right)-k^{+}\right)t}+\frac{A}{\left(k^{-}\left(0\right)-k^{+}\right)}\left[e^{\left(k^{-}\left(0\right)-k^{+}\right)t}-1\right]. \end{array}$$

An outbreak of morbidity (20) with a positive increment *k*^−^(0) − *k*^+^ > 0 can be extinguished only due to the lagging terms in (13).

In a stationary case,

(21) $$\begin{array}{c} \frac{dN_{2}}{dt}=\kappa^{-}\left|N_{2}\left(t\right)-N_{2}\left(t-\tau \right)\right|-\kappa^{+}N_{2}\left(t\right)-\kappa^{с}N_{2}\left(t-\tau \right)+А=0,N_{2}\left(t\right)=N_{2}\left(t-\tau \right). \end{array}$$

The solution, as in stationary models of laser physics with constant pumping of the active medium, takes the form

(22) $$\begin{array}{c} N_{2}=\frac{A}{\left(k^{+}+k^{с}\right)}. \end{array}$$

The stationary value (22) does not depend on  *N*_0_, *k*^−^.

Figure 1 shows epidemic curves when *N*_0_ = 6∙10^5^ a constant source of infection operates in a settlement with a population of people (a medium-sized city). Such a source can be an infected contingent arriving in a settlement with the external passenger traffic. Curve 1 corresponds to the source *A* = 10 people/day and *t*′ = 20 and *t*^″^ = 50 in coefficients (17). A later adoption of quarantine measures *t*′ = 50 and *t*^″^ = 80 with the same source corresponds to curve 2, and the outbreak is extinguished only due to the lagging terms in (13) before the quarantine measures are taken. Both curves tend to one stationary value (22) determined by the action of the source. Curve 3 corresponds to the source *A* = 50 people/day and *t*′ = 20 and *t*^″^ = 50 in the coefficients (17) and reaches a stationary value (22) 5 times greater than curves 1.2. Note that the wavy behavior to the right of the maximum is due to the complex structure of the second equation of system (13). The calculations do not depend on the value *N*_1_; this dependence can manifest itself when the entire population of the city is ill or when it is vaccinated.

The form of the morbidity curve is standard (rise-decline), qualitatively coincides with the results [5, 10, 11], and differs significantly over long periods: an asymptotic tail instead of a sharp exit to 0.

## 3. Inverse Problem of Epidemic Kinetics

To analyze the properties of the solution to problem (8)–(12), it is necessary to know the function of the real source  *A*(*t*). This function can be determined by solving the inverse problem of epidemic kinetics. In laser physics, this method is used to determine the pump function from the experimental emission spectra of the atoms of the medium. In epidemic statistics, infection rates (per dayΔ*t* = 1) and death rates (per day) are used, which correspond to the solution components (13).

(23) $$\begin{array}{c} \frac{\Delta N_{2}}{\Delta t}=\kappa^{-}\left|N_{2}\left(t\right)-N_{2}\left(t-\tau \right)\right|+А, \end{array}$$

(24) $$\begin{array}{c} \frac{\Delta N_{4}}{\Delta t}=\kappa^{с}N_{2}\left(t-\tau \right). \end{array}$$

Determination of the source of infection *A*(*t*) can be done by solving the inverse problem (8), where the left side is the statistics data [12] and the right side is the solution to system (1) with the desired source *A*(*t*). In the formulation of a direct problem, the equations and coefficients are unchanged, and only the initial population size changes. Step-by-step time fitting is used as a numerical method for solving the inverse problem.  Figure 2 shows the daily statistics of morbidity in Moscow ( *N*_0_ = 1.2∙10^7^) for the 539 days starting from 12 March 2020 (1, solid line); the source determined by solving the inverse problem (23) and (13) (2, dashed line); calculated data (23) of model (1) with the obtained source (3, points).

The average deviation of the calculation data and statistics is 629 people/day, which corresponds to a relative error of less than 7%. A wave can be understood as a maximum amplitude with a width determined at half height. Waves in the number of infected, the daily increment of the infected, and the source of infection have shifted maximum positions. The structure with source waves is primary and determined according to epidemic statistics. Two main factors for the emergence of waves of infection are as follows: the importation of infected with an external transport stream and an internal increase in contacts due to noncompliance with sanitary standards. The combination of these factors is indirectly taken into account in the source as a result of solving the inverse problem. The first wave has a maximum of 54 days of calculations (5 May 2020), a rather narrow width due to the adoption of strict quarantine measures in the form of lockdown, which are taken into account in the quasistationary mode in the source indirectly through statistical data. The second factor seems to have been predominant. The second wave, which was more extended, had a large amplitude and was formed by a combination of two factors. The development of the third wave is associated with the emergence of the Indian strain, and the decline of the wave is due to vaccination.

Figure 3 shows the curves of morbidity *N*_2_(*t*)  (solid) and lethality *N*_4_(*t*) (dotted line), calculated according to model (13) with the obtained source and the modified coefficient *k*^*с*^ = 1/200 .

The integral number of infected people in Moscow since the beginning of the epidemic of 1 September 2021 is the following: statistical data, 1,568,767 7 people; calculation data from the received source, 1,597,000 people.

Statistical data (23) and (24) in the quasistationary approximation taking into account (22) can be represented as

(25) $$\begin{array}{c} \frac{\Delta N_{2}}{\Delta t}=\kappa^{-}\left|N_{2}\left(t\right)-N_{2}\left(t-\tau \right)\right|+А\approx А, \end{array}$$

(26) $$\begin{array}{c} \frac{\Delta N_{4}}{\Delta t}=\kappa^{с}N_{2}\left(t-\tau \right)\approx \frac{k^{с}A}{\left(k^{+}+k^{с}\right)}. \end{array}$$

The quasistationary approximation is well known in the theory of laser media. Such a regime arises when the time of action of the pumping of the laser medium is many times longer than the times of depletion of the energy states of the atoms of the active medium.

Both statistics (25) and (26) are determined by the source of infection *A*. The model gives overestimated values for the lethal group, which requires correction of the coefficient *κ*^*с*^. The coefficient *κ*^*с*^is reduced by 4 times, while the residual value changes from 626 people/day to 644 people/day with the same source of infection, i.e., the dependence of the model results on the coefficient is not significant. Mortality statistics (26) cannot be used to independently determine the source of infection due to the uncertainty in the frequency of death *κ*^*с*^ .

## 4. Analysis of the Correlation between the Source of Infection and the Number of Infected *N*_2_(*t*)

The source *А*(*t*) is obtained as a result of solving the inverse problem of epidkinetics and the  *N*_2_(*t*) solution of the direct problem of epidkinetics with the obtained source.  Figure 4 shows a graph of the parametric *А*(*N*_2_)as follows: thick curve, the first wave; thin curve, the second wave; the dotted line, the third wave; curve points–stationary relation

(27) $$\begin{array}{c} A=N_{2}\left(k^{+}+k^{с}\right),\;k^{с}=\frac{1}{200\;}. \end{array}$$

The dependence is of a spiral nature, so that the values *А*, *N*_2_can be interpreted as waves, but their maxima do not coincide, i.e., the waves are different. In general, the values *А*, *N*_2_ are correlated, tend to a stationary connection, with the exception of the lower part of the graphs, where *N*_2_ decreases at constant *A*, which does not contradict the course of the incidence curve (Figure 1). Correlation *А*, *N*_2_means that the source is formed by the number of infected. Areas marked with numbers 1, 2, 3a, and 3b are highlighted, in which the source sharply increases with the number of infected.  Section 1 is a jump on the 50th day of observations (1 May 2020, a holiday in the Russian Federation). Plot 2 - smoother growth 171-202 days of observations (30 August 2020 – 30 September 2020 - the end of summer vacations and the beginning of the school year). Points 3a -393 (12 April 2021), 3b - 456 (11 June 2021). A jump to the holiday, the second factor works, 2 is a combination of factors, 3a is the second factor, and 3b is the first factor (the import of an Indian strain).

Application of the theory for other cities gives [13] for 1 September 2021 the position of the coordinate of the end point of the spiral: Berlin, *A* = 906; New York, *A* = 4126; and Catalonia, *A* = 636. Quantity information *N*_2_ is not available. Recession of the epidemic is the approach of the spiral to the origin.

## 5. Accounting for Vaccination in the Model of Epidemic Kinetics

Vaccination above is indirectly accounted for by reducing the source of infection. Direct accounting of vaccination can be performed within the framework of the following model:

(28) $$\begin{array}{c} \overset{4}{\underset{i=1}{\sum }}N_{i}\left(t\right)=N_{0},\frac{dN_{1}}{dt}\left(t\right)=-\kappa^{-}\left|N_{2}\left(t\right)-N_{2}\left(t-\tau \right)\right|-А\left(t\right)-B\left(t\right),\frac{dN_{2}}{dt}\left(t\right)=\kappa^{-}\left|N_{2}\left(t\right)-N_{2}\left(t-\tau \right)\right|-\kappa^{+}N_{2}\left(t\right)-\kappa^{с}N_{2}\left(t-\tau \right)+А\left(t\right),\frac{dN_{3}}{dt}\left(t\right)=\kappa^{+}N_{2}\left(t\right)+B\left(t\right),\frac{\;dN_{4}}{dt}\left(t\right)=\kappa^{с}N_{2}\left(t-\tau \right). \end{array}$$

This adds the vaccination rate *B*(*t*) with a minus sign to the equation for *N*_1_ and a plus sign to the equation for *N*_3_. In the stationary case, in the approximation *А*(*t*) ≈ const, *B*(*t*) ≈ const

(29) $$\begin{array}{c} \;N_{1}=N_{0}-\left(A+B\right)t;N_{2}=\frac{A}{\left(k^{+}+k^{с}\right)};N_{3}=\left(\frac{k^{+}A}{k^{+}+k^{с}}+B\right)t;N_{4}=\frac{k^{с}A}{\left(k^{+}+k^{с}\right)}t. \end{array}$$

Vaccination with this approach reduces the size of group 1, increases the number of group 3, and directly not affects the abundance and groups 2 and 4. The indirect impact of vaccination on the number of groups is obtained from (29) in the form of evaluations and infection rate with the vaccinations.

(30) $$\begin{array}{c} \kappa^{-}\sim \frac{N_{1}\left(t\right)}{N_{0}}\sim 1-\frac{\left(A+B\right)t}{N_{0}}. \end{array}$$

## 6. Reproduction Coefficient

In epidemiology, the process of epidemic development is often described using the reproduction coefficient. The rate of spread (reproduction) of virus *R*(*t*) is an indicator that determines the average number of people infected by one patient before his isolation (or recovery). It is calculated based on the data on the increase in new cases over the last *τ*_0_ days. The virus spread coefficient is used to make decisions about the transition to the next stage of lifting restrictions

(31) $$\begin{array}{c} R\left(t\right)=\frac{1}{N_{2}\left(t\right)}\frac{dN_{-}\left(t\right)}{dt}∙\tau_{0}. \end{array}$$

*N*_2_(*t*) is the number of infected persons, *dN*_−_(*t*)/*dt* is the rate of infections per day *t*, *τ*_0_ is the time of the spread of infection by an infected person, and *N*_−_(*t*) is the global statistic parameter (the number of infections since the outbreak).  Figure 5 shows the time course of the reproduction coefficient based on statistical data for the city of Moscow and the value of *τ*_0_ = *τ*^+^ = 15 days.

The graph indicates an obvious weakening of the viral infection compared to the first wave of the virus, as well as the transition of the epidemic to a quasistationary mode, where

(32) $$\begin{array}{c} R\left(t\right)\approx \tau^{+}\left(k^{+}+k^{с}\right)\approx 1. \end{array}$$

## 7. Discussion

The study of epidemic kinetics within the framework of a new theoretical model reproduces the course of the infection curve with three characteristic areas: rise, fall, and exit to a stationary value. The spread of infection is described by paired interactions with average speeds and the source of infection. The dynamic system underlying the model is nonstandard—with lagging terms and a source that is determined as a result of solving the inverse problem. The presence of a source leading to the possibility of describing the stationary mode of the epidemic distinguishes the proposed model from all other previously known ones.

The model with a source is minimal in the number of group states, which allows, with the uncertainty of the coefficients of the problem, to set and solve the inverse problem of epidemic kinetics to determine the time course of the source of infection for Moscow by one set of statistics in the form of a daily increase in morbidity. Another set of statistics is used to refine the coefficients. Next, a direct problem is solved with the found source and all the characteristics of the temporal evolution of the epidemic are obtained, including an estimate of the reproduction coefficient. Solving the direct problem of epidemic kinetics with the found source, the authors obtained a coincidence with the statistical data for the city of Moscow with an error of not more than 7%. The formulation and solution of the inverse problem of epidemic kinetics within the framework of the model under consideration is the second distinctive feature of the approach used. The first wave of the epidemic proceeds in a nonstationary mode and has the duration of 90-100 days. Further, while maintaining sanitary measures, the epidemic proceeds in a quasistationary mode, for which the source of infection is crucial. The spiral relationship of the source with the number of infected determines the dependence of the source on *N*_2_(*t*) and the wave-like nature of the epidemic development. The beginning of the rise of waves is associated with an increase in contacts and incoming traffic flow, and the decline of waves is associated with the introduction of quarantine measures. The impact of vaccination in Moscow on the reduction of the third wave is estimated as follows: mild quarantine measures reduce the level of infection by 3 times, vaccination gives an additional lowering coefficient (30), where the level of vaccination reaches values of *B*≈10^5^ person/day.

If appropriate statistical data are available, the model can be implemented for any region of the world. The data given for Berlin, *A* = 906; New York, *A* = 4126; and Catalonia, *A* = 636 are not complete in this sense. They show only one coordinate on the spiral in space (*N*_2_, *А*) at a fixed moment. The spiral connection through passenger traffic extends to other cities and regions. Individual turns of the spiral may be degenerate due to the small amplitude of the wave. The ultimate goal is to get out of the spiral to the origin:  *N*_2_ = 0, *A* = 0.

Note that our model (13)–(18) is descriptive. In order to proceed to predictions, you need to study in detail the formation of the structure of the source *A*(*t*). We hope that this part of the problem will be solved in future works.

## 8. Conclusions

The article presents a study of epidemic kinetics within the framework of a new theoretical model using kinetic elements for populations of atomic levels of an active laser medium as follows: a description of states and rates of transitions between them, an integral operator, and a source of influence on the system. In this model, the time integral operator is reduced to an algebraic form with lagging terms. It is shown that the concept of the source of infection should be used to describe a long-term epidemic. With a constant source of infection, the epidemic, in terms of the number of actively infected people, goes into a stationary mode, which does not depend on the population and the specifics of quarantine measures.

Structure of the source of quasistationary infection is not known; however, the task of describing infection statistics for a locality (city) can be solved as follows. At the first stage, the inverse problem of epidemic kinetics is solved. To determine the real source of infection, statistics were used in Moscow on the daily increase in the number of infected. At the second stage, the direct problem of epidemic kinetics with the already found source is solved. This made it possible to obtain epidemic curves that coincide with statistical data with an accuracy of 7% for the entire long-term stage of the epidemic development, taking into account three waves of infection.

The interpretation of epidemic waves generated by the source is given. Waves of infection are formed by two main factors: external incoming passenger traffic and, possibly, an increase in contacts between citizens due to the weakening of sanitary measures. In the formation of the first and third waves, an increase in contacts prevails, and in the formation of the second, a combination of factors.

It is shown that in the quasistationary mode of epidemic development, the use of two statistical data on the frequency of infection and mortality makes it possible to determine the epidemic mortality rate, which for Moscow was about 0.5% per day of the number of infected. At the same time, accurate mortality statistics cannot be used to determine the source of infection due to uncertainty in the *κ*^*с*^ mortality rate.

## Figures and Tables

**Figure 1:** Solution of system (1) with *N*_0_ = 6∙10^5^: *A* = 10, *t*′ = 20, and *t*^″^ = 50 (1); *A* = 10, *t*′ = 50, and *t*^″^ = 80 (2); *A* = 50, *t*′ = 20, and *t*^″^ = 50 (3).

**Figure 2:** Statistical data of daily morbidity in Moscow for 539 days starting from 12 March 2020 (1, solid line); the source determined by solving the inverse problem (23) and (13) (2, dashed line); calculated data of the model (1) with the obtained source (3, points).

**Figure 3:** Estimated curves of morbidity (solid) and mortality (dotted line) with the received source and the modified coefficient.

**Figure 4:** Parametric graph *А*(*N*_2_): thick curve, first wave; thin curve, the second wave; the dotted line, the third wave; points–stationary relation (9) with a coefficient *k*^*с*^ = 1/200 .

**Figure 5:** The time course of the reproduction coefficient (31) for the city of Moscow. Time *t* is specified in days.

## Data Availability

In the article, the authors used the data of the official state statistics of the Russian Federation on the incidence of COVID-19 in the city of Moscow, which are presented in link [12] and in link [13] (New York, Berlin, and Catalonia). From these data, the authors took the daily rates of infection, recovery, and mortality of citizens living in the city of Moscow for the period from the beginning of the epidemic (March 12, 2020) to the present (September 2021), which are incorporated into the presented epidemic model. The data confirming the theoretical model were also taken from the specified statistics. The calculation and statistics are close with high accuracy when the coefficient *k*^*s*^ varies.
